The article "Meta-Analysis of the Efficacy and Safety of Interleukin-23-Targeted Drugs in the Treatment of Moderate-to-Severe Psoriasis" was published in 2022. Journal: Contrast Media Mol Imaging.

# Meta-Analysis of the Efficacy and Safety of Interleukin-23-Targeted Drugs in the Treatment of Moderate-to-Severe Psoriasis

**DOI:** 10.1155/2022/2172980

**Published:** 2022-06-28

**Authors:** Teng Zhu, Lin Ma

**Affiliations:** Department of Dermatology, Beijing Children's Hospital, Capital Medical University, National Center for Children's Health, Beijing, China

## Abstract

In this study, our purpose was to systematically evaluate the efficacy and safety of interleukin-23 (IL-23)-targeted drugs in the treatment of moderate-to-severe psoriasis and provide an evidence-based reference for clinical treatment. A computer search of PubMed, EMBASE, Web of Science, Cochrane Library, Chinese Journal Full Text Database, Chinese Science and Technology Journal Database, and Wanfang Database was conducted from the establishment of the database to 2021-09-30. The efficacy of IL-23-targeted drugs (trial group) was compared with placebo (control group) in the treatment of psoriasis; i.e., PASI score improvement of 75% or more (PASI 75, PASI 90, and PASI 100) and the safety of randomized controlled trials (RCTs) were collected. Meta-analysis was performed using Rev Man 5.4.3 statistical software after data extraction for clinical studies that met the inclusion criteria. A total of 9 studies were included, all included studies were large multicenter, randomized, double-blind, placebo-controlled studies, and all used correct randomization methods and were of good quality. Meta-analysis showed that the improvement rates of PASI 75, PASI 90, and PASI 100 in the test group were superior to those in the control group (OR = 70.21 (42.25, 166.66), *P* < 0.00001), (OR = 78.41 (53.09, 115.79), *P* < 0.00001), and (OR = 77.10 (38.61, 153.99), *P* < 0.00001), *P* < 0.05. However, more adverse effects occurred, and the differences were statistically significant. IL-23-targeted drugs have significantly higher response rates compared to placebo in the treatment of psoriasis, and the safety was acceptable.

## 1. Introduction

Psoriasis, a chronic immune inflammation-mediated disease, afflicts approximately 2% of the global population [1], and the global disease burden continues to increase further [2]. The disease is most prevalent in young and middle-aged people in their 20s and 40s [3]. Not only is the disease often associated with a variety of diseases such as cardiovascular disease and metabolic syndrome [4], but it also predisposes patients to low self-esteem, depression, and anxiety, resulting in severe psychological and financial burdens [5]. The pathogenesis of psoriasis is unknown, and clinical outcomes are poor. Current research suggests that abnormal keratin-forming cell, dendritic cell and T-cell function, and excessive release of proinflammatory factors, leading to the maintenance of prolonged activation of the innate and adaptive immune systems, are important molecular pathogenic mechanisms [6]. Among these, the interleukin (IL)-23/Th-17 immune axis is a key chemotactic factor in psoriasis inflammation [7–9]. IL-23 has been shown to be an important therapeutic target in psoriasis as an upstream inflammatory factor in the IL-23/Th17 axis. IL-23-targeted drug therapy has been developed and applied clinically, but the drugs are relatively new and clinical experience is scarce. Although previous studies have summarized short-term efficacy and safety data for IL-23-targeted drugs, findings in terms of efficacy and safety remain controversial [8, 10]. Therefore, we assessed the efficacy and treatment safety of the IL-23-targeted drugs guselkumab, tildrakizumab, and rizazumab in moderate-to-severe psoriasis using a meta-analysis of all double-blind randomized, placebo-controlled trials. The effectiveness of the treatment was measured by a 75% or greater reduction in psoriasis area and severity index (PASI) scores.

## 2. Materials and Methods

This meta-analysis was conducted in accordance with the Preferred Reporting Items for Systematic reviews and Meta-Analyses (PRISMA) statement [11] and was written according to the Cochrane Handbook for the Systematic Evaluation of Interventions.

### 2.1. Inclusion and Exclusion Criteria

Inclusion criteria were as follows: clinical trials published at home and abroad, randomized, double-blind, placebo-controlled study (RCT), and the language was set to Chinese and English. Adult patients (18 years of age and older) with a clinical diagnosis of moderate-to-severe psoriasis at any treatment stage, of either gender and duration, who were not treated with biological therapy before starting IL-23-targeted drug therapy; adult patients (18 years and older) with clinically diagnosed moderate-to-severe psoriasis at any stage of treatment, regardless of gender and duration of disease, who were not on biological therapy prior to initiation of IL-23-targeted drug therapy. Patients were randomly divided into a placebo control group treated with IL-23-targeted drugs.

The proportion of patients with a 75% decrease in PASI (PASI 75) and above within the treatment cycle and the incidence of adverse reactions were used as study efficacy and safety indicators.

Exclusion criteria were as follows: (1) animal studies, pharmacokinetic and pharmacodynamic studies, case reports and review articles; (2) poor trial design or inappropriate use of statistical methods; (3) lack of data on study efficacy indicators and adverse events; (4) duplicate publications and data from the same study published multiple times over different time periods.

### 2.2. Search Strategy

In PubMed, EMBASE, Web of Science, Cochrane Library, Chinese Journal Full Text Database, Chinese Science and Technology Journal Database, and Wanfang Database, the Chinese and English literature was searched up to 2021.09.30, where the search terms in the foreign language databases were as follows: “Psoriasis ,” “Palmoplantaris Pustulosis,” “IL-23,” “Interleukin 23,” “Guselkumab,” “Secukinumab,” “Certolizumab,” “Certolizumab” “BI655066.” The search terms in the Chinese database were as follows: “psoriasis,” “psoriasis,” “rasulizumab,” “tilazumab,” “migizumab,” “IL-23,” and “interleukin-23.” There is no restriction on age, gender, or follow-up time in the search.

### 2.3. Data Extraction and Literature Quality Evaluation

Literature screening was carried out independently by an investigator based on the nadir criteria, with the second author making the final decision to exclude all other study types other than RCTs if there was a dispute. The titles and abstracts of the remaining records were then checked, and all irrelevant records were excluded. Finally, the full-text versions of the remaining records were assessed for eligibility and all studies that did not meet all specific eligibility criteria were excluded. The full text of the literature included in the evaluation was located and the literature was independently evaluated according to the normative evaluation method, and an information collection form was completed. Information extracted included the following: (1) name of the first author, year of publication, intervention, course of treatment, sample size, patient gender and mean age, duration of disease, and baseline PASI; (2) outcome indicators: 75% (PASI 75), 90% (PASI 90), and 100% (PASI 100) improvement in patient PASI scores at the end of the course of treatment and incidence of adverse events. Quality assessment was performed according to the risk of bias assessment method for RCTs recommended in the Cochrane systematic appraisal manual 5.0.

### 2.4. Statistical Analysis

Review Manager 5.4.3 software was used to analyze the data. For continuous variables, mean difference (MD) or standardized mean difference (SMD) was used as the effect analysis statistic; for categorical variables, odds ratio (OR) was used as the effect analysis statistic and 95% confidence intervals (CI) were used for interval estimation. Heterogeneity tests for the included studies were then conducted using 2-test pairs. A fixed-effects model was used if statistical heterogeneity between the studies' results was low (*P* > 0.10, I2 ≤ 50%); conversely, a random-effects model was used. And the sources of their heterogeneity were analyzed. One study at a time was removed to show the effect of a particular study on the combined effect, which in turn was excluded for sensitivity analysis. Statistical differences were demonstrated when *P* < 0.05. For the included studies, patients who received a placebo during the induction phase switched to active treatment during the maintenance phase. We assumed that the placebo effect during the induction phase continued until the end of the maintenance phase. In these studies, data from the induction phase in the placebo control group were compared with data from the maintenance phase in the treatment group.

## 3. Results

### 3.1. Literature Search Results

The literature screening process is shown in Figure 1. 10, 238 relevant articles were initially searched according to the search strategy, and 3, 261 articles were de-weighted using Endnote software. After strict inclusion and exclusion criteria were followed in a stratified manner, nine papers were finally included [12–20], covering 10 treatment groups. All the literature was in English.

### 3.2. Basic Information of Included Studies

A total of 5599 patients were included in this study, as shown in Table 1.

### 3.3. Inclusion of Methodological Quality Evaluation Results

The included studies were large multicenter, randomized, double-blind, placebo-controlled studies, and all used the correct randomization method, including computer randomization and central randomization method, with detailed instructions for withdrawal, follow-up, and loss to follow-up. Because all studies were funded by pharmaceutical companies, other biases were judged to exist, as detailed in Figure 2.

### 3.4. Meta-Analysis Results

#### 3.4.1. Efficacy Analysis

*(1) PASI 75*. All nine studies reported the results of anti-IL-23 antibodies compared to placebo for moderate-to-severe psoriasis regarding PASI 90 index, with 2292 cases (56.6%) achieving PASI 90 index at the end of the course of treatment and only 26 cases (1.7%) achieving PASI 90 index in the placebo group. The results showed that the anti-IL-23 antibody significantly increased PASI 90 attainment compared to the placebo (OR = 78.41 (53.09, 115.79), *P* < 0.01). Meta-analysis results suggested that the PASI 90 compliance rate was significantly higher in the treatment group compared to the placebo group, with a statistically significant difference (Figure 3).

*(2) PASI 90*. All nine studies reported the results of anti-IL-23 antibodies compared to placebo for moderate-to-severe psoriasis regarding PASI 90 index, with 2292 cases (56.6%) achieving PASI 90 index at the end of the course of treatment and only 26 cases (1.7%) achieving PASI 90 index in the placebo group. The results showed that the anti-IL-23 antibody significantly increased PASI 90 attainment compared to the placebo (OR = 78.41 (53.09, 115.79), *P* < 0.01). Meta-analysis results suggested that the PASI 90 compliance rate was significantly higher in the treatment group compared to the placebo group, with a statistically significant difference (Figure 4).

*(3) PASI 100*. Eight studies with nine treatment groups reported the results of anti-IL-23 antibody compared to placebo treatment for moderate-to-severe psoriasis regarding the PASI 100 index. Of the 3687 cases in the anti-IL-23 antibody treatment group, 1051 (28.5%) did not achieve the PASI 100 index during the course of treatment and only 5 (0.3%) of the 1451 cases in the placebo group achieved the PASI 100 index. The results showed that the anti-IL-23 antibody significantly increased PASI 100 attainment compared to the placebo (OR = 77.10 (38.61, 153.99), *P* < 0.01). The results of the meta-analysis suggested that the PASI 100 compliance rate was much higher in the treatment group than in the placebo group, and the difference was statistically significant (Figure 5).

#### 3.4.2. Safety Analysis

*(1) Incidence of Adverse Reactions*. Eight included literature involving 9 treatment groups reported the incidence of adverse reactions of anti-IL-23 antibody in the treatment of moderate-to-severe psoriasis. The results of the heterogeneity test showed that *P* < 0.00001 and I2 = 90%, and the statistical heterogeneity was high among the studies, so the random-effects model was used for combined analysis. The incidence of total adverse events was higher in moderate-to-severe psoriasis treated with anti-IL-23 antibody-targeted drugs than with placebo (OR = 1.66 (1.06, 2.60), *P*=0.03 (see Figure 6)).

### 3.5. Publication Bias Analysis

In this study, the PASI 75 compliance rate was the most important utility index, so PASI 75 was selected to draw an inverted funnel plot for publication bias analysis. The scatter points of each study in the figure were basically symmetrical along the center line, and basically fell within the confidence interval, indicating that there was a small possibility of publication bias (Figure 7).

## 4. Discussion

Psoriasis always occurs in young adults with no obvious difference in morbidities in different sexes. The clinical manifestations of psoriasis are mainly erythema and squama, which can be observed on the whole body, and these clinical manifestations are more common on the scalp and the extensor aspect of arms and legs. Due to the high universality of psoriasis, the WHO regarded psoriasis as a serious global problem. The molecular mechanism studies of psoriasis show that the innate and acquired immune systems remain active in the long term because the immune cells in the patient's body release proinflammatory factors excessively; thus, the long-term active state of immune systems causes persistent damage to multiple tissues and organs. Monoclonal antibodies blocking IL-23 show efficacy in adults with moderate-to-severe psoriasis, such as ustekinumab (Ust) targeting IL-12/IL-23p40 and guselkumab (Gus), tildrakizumab (Til), and risankizumab (Ris) targeting IL-23p19.

Psoriasis is a chronic disease; it would be beneficial to understand better the relative effectiveness of biological drugs rather than induction. This study was a meta-analysis comparing efficacy and safety data for IL-23-targeted drugs (guselkumab, secukinumab, and certolizumab) in the treatment of moderate-to-severe psoriasis. Previous studies [21,22] have suggested that as IL-17-targeted drugs are administered at higher doses and frequencies than biologics targeting IL-23, this may explain the better efficacy and more adverse events associated with IL-17 inhibitors. It is known that IL-17 is located downstream of IL-23 in the pathogenesis of psoriasis [23] and therefore, treatment of psoriasis by antagonizing IL-17 may be more prone to relapse than blocking IL-23, thus requiring patients to take the drug more frequently [24]. In addition, another reason why blocking IL-17 has a relatively greater impact than blocking IL-23 may be that IL-17 is essential for fighting against infections by pathogenic bacteria such as *Staphylococcus aureus* and *Candida albicans* on the skin, and therefore biologics targeting IL-23 may be a better choice for patients with psoriasis in terms of drug compliance and safety [25, 26].

In this study, based on the results of PASI 75, PASI 90, and PASI 100, we observed that interleukin-23-targeted drugs had a more significant effect on patients with moderate-to-severe psoriasis, with patients in the trial group significantly outperforming the control group in terms of improvement in PASI 75, PASI 90, and PASI 100.

Throughout the treatment period, the incidence of adverse events (AEs) was higher in each study than in the placebo group, regardless of any dose group, for those receiving IL-23-targeted drugs. The types and patterns of AEs reported were generally similar to those reported in the placebo control group. Moreover, changes in the dose of the targeted drug were not found to result in significant changes in the amount of AEs occurring. Infection was the most common AE, but serious AEs leading to treatment discontinuation were rare and there were no deaths associated with this treatment, which would suggest that the safety profile of IL-23-targeted drugs is moderate.

In terms of the overall quality of the included literature, this meta-analysis operated according to strict criteria in terms of literature inclusion and exclusion criteria, but there are some limitations to this study. (1) The number of IL-23-targeted drugs included in this article is large for tumors, and the dose and duration of treatment vary for each drug; whether this variation may cause bias in treatment outcomes has not yet been analyzed in this article. (2) This article was searched in a limited number of languages, and there may be articles in other languages that were not included, and the accuracy of the meta-analysis findings may be somewhat affected.

## 5. Conclusion

In summary, IL-23-targeted drugs can significantly improve the response rate compared with placebo in the treatment of psoriasis, with fair safety.

## Figures and Tables

**Figure 1:** Literature screening flow chart.

**Figure 2:** Methodological quality assessment of included literature trials.

**Figure 3:** Forest plot for PASI 75.

**Figure 4:** Forest plot for PASI 90.

**Figure 5:** Forest plot for PASI 100.

**Figure 6:** Adverse reactions.

**Figure 7:** Funnel plot.

**Table 1:** Basic information of included studies.

First author and year of publication	Number of subjects		Interventions		Treatment course	Baseline condition	PASI 75 (treatment group vs. control group) (case)	PASI 90 (treatment group vs. control group) (case)	PASI 100 (treatment group vs. control group) (case)	Incidence of adverse reactions (test group vs. control group) (case)
	Test group	Control group	Test group	Control group						
Blauvelt et al. [14]	329	174	Guselkumab 100 mg (0 week, 4 weeks, and then 1 time/8 weeks)	Placebo	48 w	Similar	300 vs. 10	241 vs. 5	123 vs. 1	243 vs. 86

Ohtsuki et al. [17]	128	64	Guselkumab 50 mg or 100 mg (0, 4, 8 weeks, and then 1/8 weeks)	Placebo	52 w	Similar	117 vs. 4	98 vs. 0	55 vs. 0	111 vs. 36

Reich et al. [15]	496	248	Guselkumab 100 mg (0 week, 4 weeks, 8 weeks, and then 1 time/8 weeks)	Placebo	28 w	Similar	442 vs. 20	373 vs. 6	219 vs. 2	288 vs. 111

Cai at al. [19]	331	110	Secukinumab 300 mg or 150 mg (0 week, 1 week, 2 weeks, 3 weeks, and then 1 time/4 weeks)	Placebo	52 w	Similar	305 vs. 4	256 vs. 1	128 vs. 0	298 vs. 66

Gottlieb et al. [13]	361	100	Certolizumab 400 mg or 200 mg (once/2 weeks)	Placebo	48 w	Similar	287 vs. 10	176 vs. 3	—	—

Gordon et al. [18]	981	484	Briakinumab 200 mg (0 week, 3 weeks), 100 mg (8 weeks)	Placebo	52 w	Similar	792 vs. 22	604 vs. 7	316 vs. 0	517 vs. 229

Krueger et al. [12]	31	8	BI655066 intravenous or subcutaneous injection	Placebo	24 w	Similar	22 vs. 1	15 vs. 0	9 vs. 0	20 vs. 7

Reich et al. [15]	617	155	Tildrakizumab 100 mg or 200 mg (0 week, 4 weeks, 16 weeks)	Placebo	28 w	Similar	389 vs. 9	216 vs. 4	86 vs. 2	276 vs. 74

Reich et al. [15]	621	156	Tildrakizumab 100 mg or 200 mg (0 week, 4 weeks, 16 weeks)	Placebo	28 w	Similar	394 vs. 9	234 vs. 2	75 vs. 0	291 vs. 86

Reich et al. [16]	153	52	Mirikizumab 30 mg, 100 mg, 300 mg (0 week, 8 weeks)	Placebo	16 w	Similar	105 vs. 2	79 vs. 0	40 vs. 0	74 vs. 25

## Data Availability

The datasets used and analyzed during the current study are available from the corresponding author on reasonable request.
